# Experimental Research on the Antitumor Effect of Human Gastric Cancer Cells Transplanted in Nude Mice Based on Deep Learning Combined with Spleen-Invigorating Chinese Medicine

This article has been retracted.

**DOI:** 10.1155/2022/3010901

**Published:** 2022-02-12

**Authors:** Ke Ai, Ding Yuan, Jie Zheng

**Affiliations:** ^1^Medical College, China Three Gorges University, Yichang, 443000 Hubei, China; ^2^Third-Grade Pharmacological Laboratory on TCM Approved by the State Administration of Traditional Chinese Medicine, China Three Gorges University, Yichang, 443000 Hubei, China

## Abstract

Gastric cancer is still the fifth most common malignant tumor in the world and has the fourth highest mortality rate in the world. Gastric cancer is difficult to treat because of its unobvious onset, low resection rate, and rapid deterioration. Therefore, humans have been working hard to combat gastric cancer. At present, the most commonly used treatment method is radiotherapy. However, this method will damage the normal tissues of the irradiated area while treating malignant tumor cells. It not only has side effects of damage to the patient's skin and mucous membranes but also needs high-rate radiotherapy and has high cost for chemotherapy. In order to solve these problems, it is necessary to find new treatment methods. This article proposes the use of Chinese medicine to invigorate the spleen to inhibit human gastric cancer cells. This article combines modern machine learning technology with traditional Chinese medicine and combines traditional Chinese medicine physiotherapy with Western medicine nude mouse transplantation experiments. The treatment of tumors in Chinese medicine is based on the theory of Chinese medicine and has different characteristics. Western medicine has the advantage of permanently injuring patients. The process of the experiment is to transplant human-derived gastric cancer cells into nude mice. After grouping treatments and obtaining comparative data, deep learning techniques are used to analyze the properties of Chinese medicines for strengthening the spleen and to compare the properties of Chinese medicines for strengthening the spleen. The experimental results showed that the tumor inhibition rate of mice using fluorouracil was 18%, the tumor inhibition rate of mice using low-dose Chinese medicine was 16%, and the tumor inhibition rate of mice using high-dose Chinese medicine reached 52%. 80 days after the experiment, the survival rate of mice using high-dose Chinese medicine is 100% higher than that of mice without treatment.

## 1. Introduction

### 1.1. Background

In 2020, the World Health Organization's International Agency for Research on Cancer (IARC) released the latest global cancer burden data. There are 1.92 million new cancer cases worldwide and 9.96 million deaths from cancer. At present, the academic circles have not yet reached a unified conclusion on the exact cause of gastric cancer, but with further research on the etiology of tumors, a variety of factors such as mutational, genetic, physical, and chemical carcinogenesis has been formed. Surgery, radiotherapy and chemotherapy are the traditional ways to treat gastric cancer. 50% of the treated patients will relapse, and the 5-year survival rate is only 20%. Therefore, the development of new and more effective treatments has always been an important direction in the field of basic research. In recent years, there have been more and more researches on Chinese medicine in China. In this experiment, human gastric cancer cells were transplanted into nude mice and then treated in groups and compared with the data. It was concluded that the survival rate of mice using large doses of traditional Chinese medicine was higher.

### 1.2. Significance

Many studies have shown that Chinese medicine for strengthening the spleen and active ingredients extracted from Chinese medicine may inhibit the growth of gastric cancer cells. This effect may be related to the inhibition of tumor spread, and there is a specific correlation between the two. Therefore, exploring Chinese herbal medicine for strengthening the spleen to treat gastric cancer has become a research of broad significance. Effective use of the advantages of traditional Chinese herbal medicines and modern advanced science and technology to develop effective and distinctive antitumor drugs is the current difficulty, focus, and hotspot in the field of Chinese herbal antitumor research. This study is aimed at demonstrating the effect of spleen-invigorating Chinese medicine on tumor drug-resistant cells and the effect of reversing tumor drug resistance and preliminarily exploring the mechanism of reversing drug resistance, which is of great significance for the clinical search for highly effective and low-side effect drugs. In addition, the deep learning model in this article may also be more widely used in the fields of chemistry, pharmacology, and informatics, because it helps improve the way humans predict drugs.

### 1.3. Related Work

At present, many scholars have proposed the use of anticancer Chinese medicine for clinical prevention of diseases. They reviewed the experimental research of anticancer compound prescriptions in the past 10 years and summarized the establishment of animal models, extraction of effective ingredients, discussion of tumor suppression effects, and regulation of immune function. With the progress of the society, more and more scholars have studied the transplanted tumors of gastric cancer cells in nude mice under deep learning. Hao et al. proposed that with the increase in the amount of deep learning data and computing power, neural networks with more complex structures have received widespread attention and have been used in various fields. They briefly described deep learning in the field of neural networks, including the most widely used architecture model and training algorithm. But their research did not give actual usage scenarios [1]. Yamins and Dicarlo studied the latest advances in deep learning in the broader modeling context and described some of the key technological innovations that support it and outlined how to use the goal-driven HCNN method to gain a deeper understanding of the development and organization of sensory cortex processing. But the research focuses on the field of machine learning theory, and its practicality is not strong [2]. Shen et al. proposed that machine learning is helping to identify, classify, and quantify medical images. Deep learning technology is rapidly becoming the most advanced technology. They reviewed the use of anatomy and cell structure detection, image registration, computer-aided disease diagnosis, and tissue segmentation. The shortcomings of their view on the success of deep learning is that they are more one sided, paid more attention to Western medicine, and had touched on Chinese medicine [3]. Zhang et al. combined deep learning and traditional Chinese medicine theories to explore the wisdom of Chinese medicine for the treatment of hypertension. He proposed the use of a stacked autoencoder model to divide clinical cases into different groups based on symptoms. They also discussed and summarized the effect of Traditional Chinese medicine on hypertension, the therapeutic effect of various symptoms, and reviewed the related work of deep learning model in medical application. The deficiency of the research is that the combination of deep learning and traditional Chinese medicine is not perfect [4]. Alice et al. believe that advanced artificial intelligence technology has created new opportunities for the development of digital and intelligent TCM pulse diagnosis and the exploration of the scientific basis of TCM. They discussed the artificial intelligence technology applied in TCM pulse diagnosis and its potential applications and advances in artificial intelligence technology, but their research focuses on the consultation stage and there is no solution for the physical therapy stage [5]. Zhao et al. believe that traditional Chinese medicine is an ancient subject, but it is difficult to assess whether traditional Chinese medicine physiotherapy can play an important role in the treatment of various diseases. They pointed out that the limitations of traditional Chinese medicine mainly include the limited scope of application and the need for the cooperation of traditional Chinese medicine clinicians. But he did not give a solution to the proposed limitations, only stating the problem [6]. Wang et al. studied the effect of the drug resistance of gastric cancer cells on chemotherapeutics. The results of the experiment can reduce cell viability through the synergistic effect of Sal-B and DDP. This experiment is of great significance to solve the drug resistance of tumor cancer cells, but the experimental treatment cost is too high and ordinary people cannot use the experimental results [7]. Yu et al. explored the role of traditional Chinese medicine in inhibiting tumor growth and improving the overall condition of mice in a nude mouse model of gastric cancer subcutaneous transplantation. This method can reduce the activity of gastric cancer cells in nude mice in vitro and in vivo, but this model can only treat one person at a time. Samples can be processed in batches using machine learning to achieve popularization effects [8].

### 1.4. Innovation

At present, no ideal drugs for controlling gastric tumors have been found and continuing to find low-toxic and high-efficiency drugs is an important direction and goal of the current research in the field of tumor multidrug resistance. Relying on the extensive development of artificial neural networks in recent years, deep learning technology has achieved amazing results in computer vision, speech recognition, and natural language processing. This article describes and summarizes the development process of deep learning, research status of deep learning in medicine, challenges, and shortcomings in detail. Using the deep learning framework, certain characteristics of drugs can be predicted based on the data characteristics of drugs; this article also boldly proposes that healthy *Atractylodes macrocephala*, a traditional Chinese medicine of the spleen, has an inhibitory effect on gastric cancer cells, which is demonstrated through experiments.

## 2. Deep Learning Algorithms

Deep learning is a technology of machine learning. Its definition originated from the research of artificial neural networks. Deep learning detects the performance of distributed functions of data by combining low-level features to form a more abstract and higher-level attribute category or function [9]. The purpose of deep learning is to build a neural network that simulates the human brain for analysis and learning. This is a mechanism that imitates the human brain and interprets data such as images, sounds, and texts.

Artificial neural networks are machine learning models inspired by the central nervous system. The connection between two neurons is a weighted sum of adaptive weights, which represents the advantages of input and output neurons [10]. A complete multilayer neural network, the first layer is the input layer, the input vector is the same size as the number of neurons, the second layer is the hidden layer, its neurons have nonlinear activation characteristics, the third layer is the output layer. The output of the neurons is collected by it, and finally, they are weighted and summed. Get the output formula (1) of the artificial neural network.

(1) $$\begin{array}{c} yt=f\left(\overset{n}{\underset{t=1}{\sum }}rtxt+bt\right). \end{array}$$

Among them, *f*(*x*) is a nonlinear function, *r*_*t*_ is the weight of the neural network, *x*_*t*_ neuron is the input value, *y*_*t*_ is the output value, and *b*_*t*_ is the error.

In 2006, because deep neural networks showed better learning performance, people's enthusiasm for neural networks was rekindled. Since then, deep learning has become a hot topic in the field of machine learning [11]. Deep learning algorithms are machine learning technologies based on distributed representations. Deep learning attempts to use a network structure composed of multiple nonlinear networks to learn advanced features of feature data. Commonly used deep learning models include deep belief networks (DBN), convolutional neural networks (CNN), and stacked autoencoders (SAE) [12].

### 2.1. Deep Belief Network (DBN)

DBN is a deep neural network composed of multiple layers of hidden units. Neurons in the same layer are not connected to each other. DBN can be used to extract and identify features of unsupervised learning methods. Then, we can add supervised learning algorithms such as Softmax and SVM/SVR to the deep belief network. The topology of a neural network includes the number of network layers, the number of neurons in each layer, and the way in which neurons are connected to each other. From the perspective of its topological structure, artificial neural network models can be divided into hierarchical and interconnected types. The schematic diagram of the 3-layer neural network model is compared with the schematic diagram of the 3-layer deep belief network as shown in Figure 1.

In the neural network model, since the previous signal is superimposed on the input, the reverse conduction is different from the deep confidence network, because for the input layer at time *t*, the residual error comes not only from the output but also from the hidden layer afterwards. The model is divided into two groups of unit *n* and *m*. A DBN with *t* hidden layers includes *t* weight matrices: *M*^1^, ⋯, *M*^*t*^, and *t* + 1 bias vectors: *b*^0^, ⋯, *b*^*t*^, which are the biases of the visible layer. The probability distribution represented by DBN is given by

(2) $$\begin{array}{c} R\left(n^{t},n^{t-1}\right)\in \exp\left(n^{t}b^{t}+n^{t-1}b^{t-1}+M^{t}n^{t}n^{t-1}\right.,\\ R\left(n_{i}^{k}=1,n^{k+1}\right)=\sigma \left(b_{i}^{k}+W_{i}^{k+1}n^{k+1}\right)\forall i,\;\forall k\in 1,\cdots ,t-2,\\ R\left(m_{i}=1,n^{1}\right)=\sigma \left(b_{i}^{0}+W_{i}^{1}n^{1}\right)\forall i. \end{array}$$

Compared with traditional neural networks, deep belief networks have better improvements in the pretraining and fine tuning stages [13]. In recent years, deep belief networks have been widely used in the field of information recognition, which has greatly improved the accuracy of information recognition [14].

### 2.2. Convolutional Neural Network (CNN)

The input data in the CNN first passes through the convolutional layer and the pooling layer for feature extraction and finally passes through the function of full connection and classifier and finally generates decision data composed of probabilistic correlation [15]. The activation functions sigmoid and tan*h* are the most commonly used in the CNN. The activation function is used for nonlinear mapping to increase the nonlinear feature expression of the network [16]. The function expression of the activation functions sigmoid and tan*h* is

(3) $$\begin{array}{c} f\left(x\right)=\frac{1}{1+e^{-x}},\\ f\left(x\right)=\frac{e^{x}-e^{-x}}{e^{x}+e^{-x}}. \end{array}$$

The activation sigmoid and tan*h* function curves are shown in Figure 2.

After some derivation, the sigmoid function can become tan*h*; the essence is unchanged, but the range becomes −1 to 1. In the early years, in order to create a brain-like activation method, researchers designed nonnegative, wide-boundary, and sparse bionic features. This is a more useful activation function. ReLU, also known as SoftPlus function, was originally used as a regression of positive numbers; ReLU brings the advantage of accelerating the convergence of training, and its expression is

(4) $$\begin{array}{c} \text{SoftPlus}\left(x\right)=ln\left(1+e^{x}\right). \end{array}$$

Because the CNN has more layers such as the convolutional layer and pooling layer, these algorithms have some differences. Here, we study and derive the back propagation and forward propagation algorithms in convolutional neural networks. The cost function formula (5) is the most important in forward propagation.

(5) $$\begin{array}{c} D^{t}=\frac{1}{2}\overset{t}{\underset{t=1}{\sum }}\overset{c}{\underset{k=1}{\sum }}{\left(x_{k}^{t}-y_{k}^{t}\right)}^{2}. \end{array}$$

*D* represents the cost, *t* represents the number of samples, *x*_*k*_^*t*^ represents the *k*-dimensional data of the *t*th sample, and *y*_*k*_^*t*^ is the same, but one is real data and the other is simulated data. A simple one-to-one sample can be expressed as follows:

(6) $$\begin{array}{c} D^{t}=\frac{1}{2}\overset{c}{\underset{k=1}{\sum }}\left(x_{k}^{t}-y_{k}^{t}\right)=\frac{1}{2}{\left\|x^{t}-y^{t}\right\|}^{2}. \end{array}$$

The cost function is the feedforward calculation of the last layer, and the previous one repeats the nesting for multiple layers. For example, the iterative output when fully connected can be as in formula (7). *t* represents the current layer, and *f*(*x*) represents the activation function such as ReLU.

(7) $$\begin{array}{c} y^{t}=f\left(x^{t}\right),\;\text{with }x^{t}=r^{t}x^{t-1}+b^{t}. \end{array}$$

Choosing a suitable activation function is not easy, and many factors need to be considered. The usual practice is to try them all if you are not sure which activation function is better and then evaluate on the validation set or test set. The back propagation algorithm is a commonly used algorithm in neural networks. The output of the convolution operation is also called the output feature map. This mapping is the output of the first layer or the output of the pooling layer, usually connecting multiple input matrices. The specific formula is

(8) $$\begin{array}{c} y_{n}^{t}=f\left(\underset{i\in Un}{\sum }x_{n}^{t-1}\cdot k_{tn}^{t}+b_{n}^{t}\right). \end{array}$$

*U*_*n*_ represents the input feature map set, and the feature map represents the correspondence between the levels determined by experience [17]. In the more common deep learning framework, it is generally to directly use all the inputs of the upper layer corresponding to the current convolution kernel to make a final merge, which can minimize the complexity of coding and the generalization ability of the model.

### 2.3. Stacked Automatic Encoder (SAE)

SAE is a simple feedforward acyclic neural network, which consists of the output layer, input layer, and multiple or single hidden layers [18]. The main difference between multilayer perceptron and self-encoding is that self-encoding uses its own input as output during the training process. By setting a hidden layer that is narrower than the input layer, SAE can learn certain characteristics of the input information. Therefore, this is an unsupervised machine learning technique [19].

The performance of the neural network also has the ability to estimate its own uncertainty. The neural network outputs a high degree of uncertainty where the prediction is wrong. SAE is actually a neural network composed of many sparse encoders, and the output of each layer is connected to all neurons in the adjacent input layer. The coding process of each layer is as follows:

(9) $$\begin{array}{c} A^{t}=f\left(x^{t}\right),\\ x^{t+1}=A^{t}\cdot r^{\left(t,1\right)}+b^{\left(t,1\right)}. \end{array}$$

The decoding steps are

(10) $$\begin{array}{c} A^{n+1}=f\left(x^{n+1}\right),\\ x^{t+n+1}=A^{t+n}\cdot r^{\left(n-t,2\right)}+b^{\left(n-t,2\right)}. \end{array}$$

Among them, *A*^*t*^ is the activation function of the nodes in the *t*th layer of the network, *x*^*t*^ is the weighted sum of all neuron inputs in the *t*th layer (for the *t*th layer, *x* is the input data), *r*^(*t*, *n*)^ is the weight value, and *b*^(*t*, *n*)^ is the deviation. SAE can be used to supervise and learn the output layer of a neural network. After feature learning, SAE can be trained and predicted in the neural network.

### 2.4. Restricted Boltzmann Machine (RBM)

The RBM is a typical deep learning generative model, which contains a layer of hidden variables and a layer of visible variables. The RBM is essentially an undirected probability graph model, which can be stacked to form a deeper model, and does not allow links between units in visible or hidden layers [20]. Suppose that the visible layer is composed of a set of *Xn* binary random variables, collectively referred to as *N*; suppose that the hidden layer of *Xm* binary random variables is denoted as *m*, and the joint probability distribution of the RBM is specified by the energy function as

(11) $$\begin{array}{c} R\left(n=n,m=m\right)=\frac{1}{G}\exp\left(-E\left(n,m\right)\right). \end{array}$$

The energy function of the RBM is given by

(12) $$\begin{array}{c} E\left(n,m\right)=-A^{t}n-B^{t}-{Cn}^{t}m. \end{array}$$

Among them, *A*, *B*, and *C* are the actual parameters of unconstrained subject learning. In formula (11), 1/*G* is called the normalization constant of the partition function:

(13) $$\begin{array}{c} \frac{1}{G}=\underset{n}{\sum }\underset{m}{\sum }\exp\left\{-E\left(n,m\right)\right\}. \end{array}$$

As can be seen in equation (13), the model is divided into two groups of unit *n* and *m*. The RBM model is described in the bipartite graph structure. One layer of the figure is the visible layer, and the other layer is the hidden layer. There is no connection between the two units shown in the RBM [21]. A simple RBM model is shown in Figure 3.

It can be seen in Figure 3 that the data slice needs to be transmitted to the corresponding training node first. This process is similar to the traditional big data platform. These data can also be stored in the distributed file system of the distributed storage, and then, the training is independent of each other, because each data node uses a copy of the model copy separately, and the hardware resources are allocated separately to achieve the purpose of horizontal expansion. This structure can realize some of the key features of the existing framework, including the smallest changes, the largest standard efficiency, and the most convenient expansion. For a binary restricted Boltzmann machine, the conditional probability distribution of *n* and *m* is given by the following formula:

(14) $$\begin{array}{c} R\left(n_{i}=1\;|\;m\right)=\sigma \left(n^{t}W_{i}+b_{i}\right),\\ R\left(n_{i}=0\;|\;m\right)=1-\sigma \left(n^{t}W_{i}+b_{i}\right). \end{array}$$

In short, RBM uses the efficient interaction between multilayer hidden variables and matrix parameterization to complete feature learning and achieve fast learning [22]. The object of the deep learning algorithm used in this article is the characteristics of the drug, which is specifically expressed as the value of the drug detected under some instruments.

## 3. Experimental Process of Transplanting Human Gastric Cancer Cells into Nude Mice

This article believes that Chinese medicine for strengthening the spleen can improve the immune function of the human body and treat a variety of chronic diseases. Gastric cancer is a malignant tumor that originates from the epithelium of the gastric mucosa. Most gastric cancers are adenocarcinomas. They have no obvious early symptoms or nonspecific symptoms such as upper abdominal discomfort and belching. They are usually similar to the symptoms of chronic gastric diseases, such as gastritis and gastric ulcers. Therefore, it is often ignored by patients. At present, the early diagnosis rate of gastric cancer is still low, and the harm is very serious. The advantages of biological models are mainly reflected in the following aspects: strong three-dimensional effect and large visibility. The structure of the organism is more complicated.  Table 1 shows the detailed cancer incidence and mortality.

### 3.1. Target Virus Construction

Nude mice are born without hair and thymus. They lack T cells and immune function, so they do not reject xenotransplanted tumors or cells. Therefore, research in various fields such as oncology, toxicology, and immunology has been widely used [23]. In clinical and laboratory research on gastric cancer, animal models are important tools for studying the mechanism of drug action on pathogens. Observing, recording, and analyzing the intervention effects of various interventions on transplanted tumor animal models is important for finding effective treatments. The human gastric cancer cell line used in the experiment was purchased from Shanghai Zhongqiao Xinzhou Biotechnology Co. Ltd. Experimental animals were 50 nude mice, 3 to 5 weeks old, purchased from Beijing Weitong Lihua Experimental Animal Co. Ltd. Then, prepare some common spleen-invigorating drugs, American ginseng, astragalus, and *Atractylodes macrocephala*. The bottle culture is in the screening and culture stages of strains, and the culture conditions should be as close as possible to the culture conditions of fermentation production.

Use sterilized culture flasks (specification: 50 mL) for culture. Place the experimental culture medium consisting of human gastric cancer cells and a high-sugar solution containing 20% calf serum in a special culture flask, and place it at a temperature of 37°C and a CO_2_ content of 5%. According to the experimental requirements, it will be cultivated at constant temperature and humidity. It was carried out in an incubator and passaged every 3 days, and logarithmic proliferation cells were collected for experiments. Human gastric cancer cells were digested with trypsin to prepare a single-cell suspension, and the cell concentration was adjusted to 0.5 × 10^6^ cells/mL under a microscope. By transplanting human CD34+ hematopoietic stem cells or PBMC into immunodeficient mice, each nude mouse was injected with 0.2 mL cell suspension subcutaneously in the right forearm and the immunodeficient mice were inoculated with human gastric cancer cell lines and then humanized mice. The model was inoculated with CDX, and the subcutaneous tumor nodule with a long diameter of 8 mm was used as the tumor formation standard to establish a nude mouse human gastric cancer transplantation tumor model. This type of model not only provides an immune microenvironment similar to the growth of human tumors but also solves the problem that the traditional CDX model of gastric cancer cannot be used to evaluate antitumor-immune agents in immunodeficient mice. The flow chart of CDX model construction is shown in Figure 4.

Ten days after modeling, 8 nude mice were randomly selected and sacrificed by spinal cord dislocation. Nude mice were transplanted with tumor tissue blocks according to the experimental requirements, and the experimental histopathological sections were observed under a light microscope: a variety of different sizes and shapes can be seen under the light microscope. Human gastric cancer cells with irregular structures and abnormal nucleus-to-cytoplasm ratios proved the success of the modeling. The data recorded below uses statistical analysis. The data is expressed in the form of mean ± standard deviation (*M* ± *S*). The comparison of means between multiple groups is performed by one-way analysis of variance. The SNK method is used to compare any two groups. When *P* < 0.05, there is statistical significance.

### 3.2. Group Treatment Experiment

In recent years, the relationship between Chinese medicine and cancer and the research on Chinese medicine for invigorating the spleen have attracted widespread attention. Chinese medicine's antitumor mechanism is very complicated. According to existing research results, the mechanism of antigastric tumors of Chinese medicine for strengthening the spleen may involve the following aspects: dehydroepiandrosterone compound inhibits tumor cells, induces cancer cell apoptosis, and promotes DNA damage repair, antioxidation, and free radical scavenging. The dosage of the medicine has nothing to do with the weight, so there is no need to set the weight group. In the experiment, nude mice were randomly divided into four groups: model control group, fluorouracil group, high-dose Chinese medicine group, and low-dose Chinese medicine group, with 12 mice in each group. The dosage of traditional Chinese medicine is converted according to the dosage of *Atractylodes macrocephala* in the “Chinese Pharmacopoeia” and the “Human and Animal Weight Conversion Formula” of the pharmacological experiment method (*dB*(g/kg) = *dA* × *RB*/*RA*) × (*WA*/*WB*) 1/3). The current adult clinical dosage is based on 60 kg as a reference. Therefore, the standard dose of *Atractylodes macrocephala* is 0.01 g/(kg · *d*), the standard dose of fluorouracil is 0.125 g/(kg · *d*), and the average body weight of nude mice is 20 g; the standard dose of *Atractylodes macrocephala* is 0.2 mg/(only · *d*); for fluorouracil, the standard dose is 2.5 mg/(only · *d*). Fluorouracil, a pyrimidine analog, is a kind of antimetabolite and is mainly used to treat tumors. The experimental dose adopts the standard dose of *Atractylodes macrocephala* as the low-dose standard, and the high dose of *Atractylodes macrocephala* is twice as high. The standard dose of *Atractylodes macrocephala* is made into 0.2, 0.4 mg/mL water-soluble quasidose, and the current concentration is 1.25 mg/mL aqueous solution. Take 2 mL and inject into the abdominal cavity after 1 day, 1 week, and 2 weeks. For the model control group, gavage 2 mL of distilled water once a day from 9 : 00 to 10 : 00 for a total of 21 days. SPSS software ranges from the description of basic statistical characteristics to various high-level analyses such as nonparametric tests and survival analysis. In addition, SPSS also has powerful drawing functions.

After 21 days of administration, the tumor volume of nude mice was measured every 3 days after administration and the average tumor volume of each group was calculated. Seven nude mice of each group were randomly selected and sacrificed. The tumors were quickly stripped and weighed. And place them in 5% paraformaldehyde solution for fixation and make pathological sections according to groups, measure the long diameter (*x*) and short diameter (*y*) of the transplanted tumor in nude mice, according to *V* (mm^3^) = 0.5 × *x* (mm) × *y* (mm)^2^ formula to calculate the volume, and repeat 3 times to measure the volume of each tumor; the recorded data are shown in Table 2.

Draw the growth curve of the transplanted tumor according to the volume record table; see Figure 5.

According to the formula to calculate the tumor inhibition rate [24], tumor inhibition rate = (the mean tumor mass of the control group − the mean tumor mass of the administration group)/the mean tumor mass of the control group × 100%. Then, the tumor inhibition rate of each group was calculated according to the formula shown in Table 3.

For the authenticity of the experimental results, the injection method is adopted, which has the least consumption of drugs, and humans can also use this method. Observe the survival period of the remaining 5 nude mice in each group. When all the nude mice in one group died, the number of nude mice living in all groups was counted and the survival rate of each group was calculated. After 80 days of observation, all mice in the high-dose Chinese medicine group survived; 2 and 3 mice survived in the fluorouracil group and low-dose Chinese medicine group, respectively; no mice survived in the model control group. Draw the survival curve of mice in each group according to the recorded information; see the Figure 6.

### 3.3. Training of the Deep Learning Classification Model

Through the above experiments, we have obtained some data that we need but it is obviously not enough to rely solely on the amount of data to draw conclusions about inhibiting cancer. Based on these data, deep learning can be performed. It attempts to model high-level abstraction of data using multiple layers of neurons composed of complex structures or nonlinear transformations, using machine analysis and simulation, and can use deep learning frameworks to compare drug property prediction. The rapid development of artificial intelligence technology provides powerful tools for analyzing large amounts of data, helping doctors make better clinical decisions, and even replacing human judgment in medicine [25]. At present, deep learning has been applied in the medical field to provide auxiliary diagnosis ideas and improve accuracy.  Figure 7 is the current application scenario designed by other scholars.

In order to better understand which molecular characteristics represent that the spleen-invigorating traditional Chinese medicine can inhibit gastric cancer, this article assumes that the samples are divided into two types, labeled as “drug toxicity positive” and “drug toxicity negative.” These two types of samples are presented in the dataset. In normal distribution, *t*-test is performed on the sample data and the obvious differences between the drug description characteristics of positive drugs and negative drugs are identified. Samples with positive and negative drug toxicity can be distinguished by their respective structural feature combinations. This shows that the structural features of these combinations are useful for prediction when predicting certain properties of drugs [26]. Studies have shown that multiple combinations of FMF (molecular structure), complexity FC (representing system complexity), and Zagreb index (representing the sum of the square of the atomicity values of all heavy atoms) are very effective in identifying positive samples [27]. The specific structural characteristics are shown in Figure 8.

It can be inferred from this whether the molecular structure of the drugs and their combination will cause harm to the human body. Therefore, they can be used in the physiotherapy task of invigorating the spleen. According to the above figure, the accuracy can be recorded as Table 4.

The 125 spleen-invigorating ingredients provided by the “Chinese Pharmacopoeia” are used as an independent test set to evaluate the classification model [28]. Among them, there are 51 drug components with good permeability of gastric cancer cells. The Tanimoto similarity (TS) of all drug components in the independent test set is calculated to evaluate whether the compounds in the independent test set contain different structures. Most compounds in the independent test set have different structures, and the diversity of structures ensures the stability of the evaluation classification model. The similarity calculation result is shown in Figure 9.

The compounds in the independent test set are structurally different from each other, and this structural diversity ensures the stability of the evaluation classification model [29]. Based on the method of mutual verification, the performance parameter area identified under the AUC curve and ROC curve scores is used. As shown in Figure 10, the deep neural network model in this paper has a high AUC score on both the test set and the independent verification set.

This section mainly introduces the knowledge of relevant network layers and the formula training derivation of convolutional neural networks that perform well in the field of medical feature classification. Although convolutional neural networks perform well in feature classification, as the amount of data increases and accuracy requirements improve, it is necessary to continuously deepen the network model, which causes the difficulty of training “gradient explosion.” For drug properties, a large dataset encoding method is used to minimize information loss. At the same time, this article proposes to use a deep learning model to predict the specific properties of drugs and small-molecule compounds. This model is better than previous drug prediction models, mainly due to deep learning, the powerful learning ability of the model [30]. When 125 drugs are used to train the deep learning combination model, the external validation data composed of 51 drugs shows that the prediction accuracy of the model is 78.8%, the sensitivity is 79.5%, the specificity is 82.4%, and the AUC value is 0.966. The data shows that the result is relatively good.

## 4. Discussion

The role of analogy is “from this to the other.” If you regard “this” as the premise and “the other” as the conclusion, then, the process of analogy thinking is a process of reasoning. Through analogy experiments, this article can also know that Chinese medicine can inhibit tumors. Although the method in this paper has excellent classification performance, there is still room for improvement in prediction accuracy. The data used to train and test the model in the experiment is collected from different research and different experimental environments. These changes will cause errors in the model and ultimately reduce the classification performance. Therefore, data obtained in larger external datasets and sophisticated experimental environments will be more useful. The antitumor method proposed in this article has the characteristics of traditional Chinese medicine and plays a prominent role in the functions of the various tissues and organs of the patient's body. The quality of life and survival time of patients with gastric cancer have been greatly improved and prolonged. In addition, if the visible tumor is removed by surgery, it does not mean that there is no residual cancer. Therefore, it is recommended to use traditional Chinese medicine with long-term postoperative treatment. Cancer cannot be completely cured by any medicine. The best way to control it is Chinese herbal medicine.

## 5. Conclusions

Analyze the objective existence of spleen deficiency caused by colorectal cancer at the cellular level. The method of invigorating qi and strengthening the spleen and anticancer can improve the spleen function of experimental nude mice with colorectal cancer. The mechanism is to increase the spleen weight and spleen coefficient and enhance the expression of splenic PKC activity. Nude mice with long-term injection of the Chinese medicine *Atractylodes macrocephala* into the abdomen grew the slowest, followed by nude mice using the Western medicine fluorouracil; the average tumor mass of nude mice injected with the *Atractylodes macrocephala* long term into the abdomen was 1.07 g, the smallest among the four groups. The tumor inhibition rate of mice using high-dose Chinese medicine reached 52%, followed by mice using fluorouracil and low-dose Chinese medicine; all mice in the high-dose group survived 80 days after the experiment, and other groups had varying degrees of the number of deaths, especially the mice in the no-treatment group; all died one after another. As long as humans take oral Chinese medicine for strengthening the spleen, it can inhibit and kill the living cells of gastric cancer and have a therapeutic effect on tumors.

## Figures and Tables

**Figure 1:** Comparison of the neural network model and deep belief network model.

**Figure 2:** Comparison of two function graphs.

**Figure 3:** An RBM drawn in the form of a Markov network.

**Figure 4:** CDX model construction process.

**Figure 5:** Comparison of the tumor growth rate and weight in each group.

**Figure 6:** Survival curves of nude mice in each group.

**Figure 7:** Deep learning applied to the medical field.

**Figure 8:** Different index combinations for drug utility discrimination.

**Figure 9:** Tanimoto similarity histogram.

**Figure 10:** ROC curve and AUC score of the validation set of negative and positive drugs.

**Table 1:** Cancer incidence and mortality in 2020.

Type	Incidence [%]	Mortality rate [%]
Breast	11.7	6.9
Lung	11.4	18.0
Colorectum	10.0	9.4
Prostate	7.3	3.8
*Stomach*	*5.6*	*7.7*
Liver	4.7	8.3
Cervix	3.1	3.4
Oesophagus	3.1	5.5
Thyroid	3.0	3.1
Bladder	3.0	3.1

**Table 2:** The volume of each group of tumors at all measurement time points (mm^3^).

	Control group	Fluorouracil	High dose	Low dose
0 d	663.92	643.81	690.21	656.36
3 d	914.73	886.54	887.87	927.03
6 d	1171.10	1106.23	1114.05	1102.27
9 d	1606.39	1591.61	1264.76	1638.67
12 d	2248.04	1727.96	1255.78	1818.27
15 d	2702.45	2050.30	1297.75	2171.78
18 d	3067.16	2391.78	1335.61	2365.02
21 d	3169.89	2594.31	1516.70	2653.29

**Table 3:** Influence of tumor weight and tumor suppression rate.

Group	*n*	Tumor weight (g)	Tumor inhibition rate
Control group	7	2.24	
Fluorouracil	7	1.83	0.18
High dose	7	1.07	0.52
Low dose	7	1.87	0.16
F		8.054	3.259
P		<0.05	<0.05

**Table 4:** Simple combination of molecular features to predict drug toxicity.

Feature combination	Accuracy (%)
Daily dose/200 + FMF/0.5 ≥ 1	82.3
Daily dose/150 + FC/200 ≥ 1	78.5
Daily dose/100 + Zagreb/200 ≥ 1	79.8
Log*P*/(20) + FMF/0.5 ≥ 1	81.7
FC ≥ 200 or FMF ≥ 0.5	80.6

## Data Availability

No data were used to support this study.
